RETRACTED

# Clinical Study of Mobile Application- (App-) Based Family-Centered Care (FCC) Model Combined with Comprehensive Iron Removal Treatment in Children with Severe Beta Thalassemia

**DOI:** 10.1155/2022/4658709

**Published:** 2022-08-05

**Authors:** Yuke Chen, Xiuping Huang, Qingmei Lu, Jian Lu, Xiaoxiao Huang, Yanni Luo, Fengxing Huang

**Affiliations:** ^1^Department of Pediatric, Affiliated Hospital of Youjiang Medical University for Nationalities, Baise 533000, China; ^2^School of Nursing, Youjiang Medical University for Nationalities, Baise 533000, China; ^3^Center for Reproductive Medicine, Affiliated Hospital of Youjiang Medical University for Nationalities, Baise 533000, China; ^4^Outpatient Department, Affiliated Hospital of Youjiang Medical University for Nationalities, Baise 533000, China

## Abstract

**Methods:**

A retrospective study was conducted on the clinical records of 148 children diagnosed with severe beta thalassemia who were admitted to our hospital between October 2018 and September 2021. The patients were separated into two groups, a control group and an intervention group, with 74 cases in each group, according to the various care approaches. The basic treatment regimen was given to all of the children: deferoxamine mesylate combined with deferiprone. During treatment, the control group received routine care, and the intervention group adopted the FCC model based on a mobile app. The quality of life scale for children and adolescents (QLSCA) score, the family assessment device (FAD) score, the exercise of self-care agency scale (ESCA) score, and the medication compliance scale score were compared between the two groups.

**Results:**

The QLSCA score, ESCA score, and medication compliance scale score of the intervention group were significantly higher than those of the control group and showed a significant difference (intergroup effect: *F* = 198.400, 259.200, and 129.800, all *P* < 0.001). Scores in both groups increased over time (time effect: *F* = 19.350, 40.830, and 12.130, all *P* < 0.001), and there was an interaction effect between grouping and time (interaction effect: *F* = 3.937, 12.020, and 5.028). The *P* values were 0.020, <0.001, and 0.007. The FAD score of the intervention group was significantly lower than that of the control group (intergroup effect: *F* = 177.200, *P* < 0.001). The FAD scores of both groups decreased over time (time effect: *F* = 7.921, *P* = 0.005). There was an interaction effect between groups and time (interaction effect: *F* = 5.206, *P* = 0.006).

**Conclusion:**

The application effect of the mobile app-based FCC model combined with the comprehensive iron removal treatment program in children with severe beta thalassemia is significant, which can significantly improve the quality of life, family function, self-care ability, and medication compliance of children, and has high clinical application value.

RETRACTED

## 1. Introduction

Thalassemia is a recessive genetic disorder characterized by the suppression of globin chain synthesis caused by a malfunction or deletion of globin genes, resulting in a change in hemoglobin composition [1]. In Baise, Guangxi, China, hemoglobinopathy is the first birth defect, and the incidence of severe *β*-thalassemia is up to 1‰ [2]. Iron overload due to transfused iron and increased iron absorption, the latter mediated by inhibition of the iron regulatory hormone hepcidin, is a common complication in people with *β*-thalassemia major, which leads to inefficient erythropoiesis and chronic anemia. Heavy beta thalassemia has a prolonged time of treatment, and the illness causes complications repeatedly. In general, infants born during the first stage of the disease display no clinical symptoms. However, between 3 and 6 months of birth, children may develop life-threatening symptoms such as hemolytic anemia, hepatosplenomegaly, low body resistance, growth retardation, and a particularly poor appearance [3]. Most children need long-term drug treatment and medical care after discharge, so the family is an important place for children to recover. However, there are still many nursing problems in the process of family care, and the caregivers of children lack relevant professional knowledge [4]. Therefore, children with severe beta thalassemia require immediate and effective nursing assistance.

Family-centered care (FCC) is a medical care strategy based on a cooperative connection between medical service providers, patients, and their mutually beneficial families. It emphasizes the role of the family in the treatment and rehabilitation of children, encourages the participation of children and their parents, and collaborates with medical staff to jointly promote children's health. It is an effective mode of pediatric nursing [5]. Currently, the FCC model has not been applied to children with thalassemia. To improve the quality of life for children, it is vital to investigate the influence of FCC on the treatment of thalassemia in children. However, due to economic constraints, most children with severe beta thalassemia cannot receive specialized guidance from medical personnel in urban areas for a long time. Therefore, the FCC requires the support of Internet technology.

This study developed a mobile app based on the Omaha System to identify health issues in children with severe beta thalassemia at home, provide reasonable therapies based on evidence, and produce a mobile app based on this knowledge. The FCC mode of three-tier A hospital-primary hospital-family connection, which was mediated by grassroots health institutions or school doctors, was also developed using the mobile app, and the effect was assessed. This mode included technology transfer, remote diagnosis and treatment, and home visits.

RETRACTED

## 2. Materials and Methods

### 2.1. General Demographic Characteristics of the Patients

The clinical data of children with severe beta thalassemia admitted to our hospital between October 2018 and September 2021 were analyzed retrospectively. Inclusion criteria are as follows: severe beta thalassemia was determined according to Rome III diagnostic criteria [6], ages 6 to 14, no contraindications for treatment in this study, and good compliance. Exclusion criteria are as follows: the presence of health-related diseases affecting the quality of life, such as chronic diseases (asthma, congenital heart disease, chronic kidney disease, cancer, etc.) and neurodevelopmental disorders (autism, epilepsy, behavioral disorders, etc.); the affected child is generally in poor health or has been exposed to serious negative events such as the death of a family member or a traffic accident in the past six months, a history of thoracic and abdominal surgery, complications with a malignant tumor and infectious diseases, and liver and kidney insufficiency. There were a total of 148 cases, comprising 78 males and 70 females. The average age was 5.46 ± 1.23 years, with a range of 6 to 12 years. The course of the disease ranged from 1 to 5 years, with an average of 3.33 ± 0.89 years. The body weight was 21.67 ± 8.75 kg. Stage of iron overload degree is as follows: IIA 43 cases, IIIA 55 cases, and IIIB 50 cases. Serum ferritin at discharge was 2539.75 ± 624.13 *μ*g/L.

### 2.2. Basic Treatment

Following their hospitalization, all of the children received complete iron removal treatment (deferoxamine mesylate with deferiprone). Specific methods are as follows: oral deferidone tablets (Apotex Inc., Registration Number H20140379, specification: 0.5 g), 75 mg/kg each time, 3 times a day, and dermal injection of deferoxamine mesylate (Wasserburger Arzneimittelwerk GmbH, Registration Number H20170147, specification: 0.5 g), 5 d/week, once/d, 40 mg/kg each time, with the portable infusion pump utilized for continuous and gradual infusion for 8-12 h. All patients were treated for 12 weeks.

### 2.3. Control Group Care Method

The control group implemented routine nursing, specifically telephone follow-up after discharge. Specific methods are as follows: within 1 week after discharge, the responsible nurse conducted a telephone follow-up for the children once. During the 4th, 8th, and 12th week after discharge, the nurse in charge continued to follow-up with each child by telephone once, understood their recovery status, and provided routine guidance, requesting that children and their parents contact the pediatric department of the hospital whenever they experience difficulties.

RETRACTED

### 2.4. Intervention Group Care Methods

Based on the control group, the intervention group implemented a mobile app-based FCC model. Specific measures include the following: (1) establishing a professional guided intervention team. Establish professional guidance and consulting team consisting of 2 chief physicians, 2 chief superintendent nurses, 1 deputy chief nurse, 3 supervisor nurses, and 3 nurses before the nursing begins. There is 1 doctor, 2 nurses, or 2 medical staff at the village health facility in the registered community or township of the child and 1 school doctor at the school where the child is enrolled. (2) Professional education is as follows. All team members received training from the Baise Health and Family Planning Commission and passed the evaluation, which included health management knowledge and technology and intervention plan needs. (3) On the day the child was discharged, the practitioner assisted poor families in installing the mobile app center type nursing home end while also teaching parents how to use the mobile app. Simultaneously, the patient's discharge information will be transferred to the primary health service station where the patient lives via the medical terminal to interact with other appropriate medical staff (the medical personnel's mobile phone installed medical micro platform). (4) Community health care personnel should visit the children within one week of their hospital discharge, with supervision content including an assessment of the environment (income, health, and shelter), physical function, psychosocial status, health behavior, and the cognition of the child and its parents, as well as targeted guidance to the children and their parents. If the children and their parents encounter difficulties, they can use the mobile app to contact the medical staff at grade A hospital for support and assistance. (5) Basic health service professionals continue to visit the children at home on the 4th, 8th, and 12th weeks after they were discharged from the hospital to understand their compliance behavior and to conduct medication guidance, care guidance, and health behavior inspection and supervision. Children and their parents can contact medical personnel at any time via a mobile app and apply for remote diagnosis and treatment. (6) Implementing FCC intervention via network mobile app: nurses provide online counseling services. Every week, a senior nurse in charge is designated as the WeChat group manager. She used the app every day from 8 : 30 to 09 : 30 and 16 : 30 to 17 : 30 to conduct online consultations for family members, answer queries, provide extensive instructions, and conduct weekly assessment of children's quality of life and implementation of nursing interventions with a specific focus. Team members received feedback from parents through communication. Parents provided feedback on their children's food, activities, quality of life, and other information to the WeChat group in the form of photographs or videos, allowing team members to intuitively evaluate the children's circumstances and deliver more targeted health education. Every week, team members used pictures, documents, videos, and other formats to spread awareness about poverty and provide popularization knowledge for children and encourage family involvement. Parents communicate with one another, share care experiences, and offer emotional support. The team members disclosed relevant information. To increase the ability of family members to care for themselves at home, team members provided hospital information on the app regularly, such as presenting “Home for the Poor” and “International Day for the Poor” health lectures.

RETRACTED

### 2.5. Observational Index

All of the study's outcomes were assessed at discharge (before intervention), 12 weeks after discharge (12 weeks after intervention), and 24 weeks after discharge (24 weeks after intervention). (1) The quality of life scale for children and adolescents (QLSCA) [7] was used to assess the quality of life, which is suitable for the multidimensional evaluation of the quality of life of primary and secondary school students aged 6-18, including 13 dimensions: self-satisfaction, teacher-student relationship, body feeling, peer relationship, parent-child relationship, exercise ability, learning ability, attitude, self-concept, emotional state, work attitude, activity opportunity, and convenience of life. Each dimension was composed of four factors: social psychological function, physical and mental health, living environment, and life quality satisfaction. Each item on the scale received four grades, giving a total score ranging from 49 to 196 points. The greater the quality of life, the higher the score. (2) The self-care ability assessment scale (ESCA) [8] was used to evaluate the ability of parents to care for their children. The scale contained 43 items across 4 dimensions, including nursing abilities, health knowledge level, self-concept, and responsibility of care, and utilized a 5-level scoring system. The total score ranged from 0 to 172, and the higher the score, the better the nursing ability. (3) The medication compliance scale [9] was used to evaluate the medication compliance of children, which included the following 10 items: forget to take their medicine behavior, change medication timing behavior, self-discontinuation of medication behavior, reducing the frequency with which medications are taken, reducing the dose behavior, taking drugs without a doctor's recommendation, using traditional Chinese medicine (TCM) or folk prescription drug behavior, according to the doctor's advice specified drugs behavior, taking the medication regularly following the doctor's recommendation behavior, and quantitative drug following the doctor's counsel behavior. Positive items comprised items 1 to 7, while negative items comprised items 8 to 10. Each item was assessed on a 5-point scale, with higher scores indicating greater drug compliance behavior. (4) The family assessment device (FAD) scale [10] was used to assess family function, which included 60 items separated into 7 components: problem-solving, communication, role, emotional response, emotional engagement, behavior control, and total function. The overall score of the scale is the average of all subscale scores. Using the grading system, 1 point signifies healthy and 4 points represent unhealthily.

RETRACTED

### 2.6. Statistical Methods

SPSS 17.0 statistical software was used to analyze the data, and the measurement data that conformed to a normal distribution were represented as “$\overset{¯}{x}\pm s$”. *T*-test was performed for comparison between the two groups, and repeated measures analysis of variance was used for comparison of data at different time points between groups. The counting data was represented by *n* (%), and a *χ*^2^ test was performed. When *P* < 0.05, the difference was considered statistically significant.

## 3. Results

### 3.1. General Demographic Characteristics of the Patients

There were a total of 148 cases included. All patients were separated into a control group and an intervention group (each containing 74 patients) based on their respective care methods. There were no statistically significant differences between the two groups in terms of gender, age, disease course, body weight, stage of iron overload degree, and serum ferritin at discharge baseline (*P* > 0.05), showing that they were comparable.  Table 1 displays the general demographic characteristics of the patients for both groups at discharge.

### 3.2. The QLSCA Score, ESCA Score, and Medication Compliance Scale Score

The QLSCA score, ESCA score, and medication compliance scale score of the intervention group were significantly higher than those of the control group, indicating a significant difference (intergroup effect: *F* = 198.400, 259.200, and 129.800, all *P* < 0.001). Scores in both groups showed a trend of increasing over time (time effect: *F* = 19.350, 40.830, and 12.130, all *P* < 0.001), and there was an interaction effect between grouping and time (interaction effect: *F* = 3.937, 12.020, and 5.028). The *P* values were 0.020, <0.001, and 0.007, respectively. The QLSCA score, ESCA score, and medication compliance scale score are provided in Tables 2–4 and Figures 1–3.

RETRACTED

### 3.3. The FAD Score (Total Function) of the Intervention Group Showed a Lower

The intervention group's FAD score was drastically lower as compared to the control group (intergroup effect: *F* = 177.200, *P* < 0.001). The FAD score of both groups decreased over time (time effect: *F* = 7.921, *P* = 0.005). There was an interaction effect between groups and time (interaction effect: *F* = 5.206, *P* = 0.006) (Table 5 and Figure 4).

## 4. Discussion

Currently, there is no effective treatment for severe beta thalassemia; however, regular blood transfusions and iron removal are used clinically to prolong the lives of children. Despite these interventions, it is still difficult to avoid direct death due to liver and kidney damage as well as heart failure before puberty [11]. The majority of children with thalassemia major require long-term drug treatment and medical care after they are discharged from the hospital because the disease has a prolonged treatment course, repeated conditions, and many complications. As a result, most of these children spend their time recovering with their families and in their communities [12]. At the same time, due to the cost burden, a lack of health resources, and other issues, most children are hospitalized when the disease worsens and then discharged to home care once the disease is cured. There are still many nursing issues in the process of family care, and caregivers such as family members of children lack essential professional skills. As a result, children require immediate assistance from nursing professionals. Children with severe thalassemia have a clear and urgent need for home care assistance. Medication guidance, health consultation, nutrition guidance, psychological nursing, disease observation, and other services are among those required [13].

This study investigated the impact of a mobile app-based FCC model in conjunction with a comprehensive iron removal treatment on children with severe beta thalassemia. Following the completion of the basic treatment of the comprehensive iron removal treatment plan, the children in the two groups received routine care and app-based FCC mode intervention, respectively. The findings demonstrated that the QLSCA score, ESCA score, and medication compliance scale score all increased, while the FAD score decreased for the children who received intervention based on the app-based FCC model. This suggests that the app-based FCC model can improve the children's quality of life, family function, self-care ability, and medication compliance. The FCC is a medical service provider based on a cooperative relationship between the patient and the family health care plan that is mutually beneficial. Its primary objective is to support children, families, and medical professionals. It highlights the importance of family care in the rehabilitation of children with the disease and encourages children and parents to participate, work with medical staff, and improve children's health [14]. The fundamental aspects of this care are respect and dignity, support for information, cooperation, and participation. Numerous practices have demonstrated that FCC may effectively improve the physical and psychological health of children and their parents, as well as their medical experience, and it has been considered the greatest kind of pediatric treatment in western countries [15, 16]. In this study, this model was applied to the care of children with thalassemia, which, along with the findings of earlier research, can aid in the recovery of children's health. Numerous studies consider FCC to be the most suitable nursing approach for pediatric patients, as it has been widely promoted and adopted abroad. Some domestic children's hospitals are planning to use it in clinical practice, education, and practical application as well [17]. The FCC model is a nursing development trend that emphasizes the importance of paying more attention to the impact of family on children's health and considering children as members of the family. In addition to curing the disease and improving the quality of life of the children, this mode of care was aimed at restoring the psychological and social functions of the children, so that they are in a normal functional state, and family members are regarded as important guardians of the children's health [18]. FCC mode is systematic and holistic care. The FCC center focuses not just on children with physical diseases but also children and families. In the process of nursing, it is necessary to evaluate all aspects of children's medical issues, including their physical, psychological, and social states, as well as their relationships with family members. In addition, it offers patients and their families educational support and complete health care [19]. Several studies have demonstrated that the implementation of FCC's medical care model in pediatric wards can not only increase the satisfaction of doctors, nurses, and patients with nursing work, improve work efficiency, and increase social recognition of medical staff but also decrease the incidence of medical errors [20]. Due to the limited sample size of this study, there is a possibility of bias in the results, which must be confirmed by studies with higher sample sizes.

RETRACTED

## 5. Conclusion

In conclusion, the mobile app-based FCC model in conjunction with comprehensive iron removal therapy has a large application effect in children with severe beta thalassemia, which can considerably enhance their quality of life, family function, self-care ability, and medication compliance. It has significant clinical use. There is a chance of some bias in the result data, which must be proven by larger sample size research. Because this study utilized a small sample size, additional research with larger sample sizes is required.

## Figures and Tables

**Figure 1:** Comparison of QLSCA score between the control and intervention groups. *n* = 74; ^∗∗^*p* < 0.01. ns: not significant.

**Figure 2:** Comparison of ESCA score between the control and intervention groups. *n* = 74; ^∗∗∗^*p* < 0.001. ns: not significant.

**Figure 3:** Comparison of medication compliance scale score between the control and intervention group. *n* = 74; ^∗∗^*p* < 0.01 and ^∗∗∗^*p* < 0.001. ns: not significant.

**Figure 4:** Comparison of FAD score (total function) between the control and intervention group. *n* = 74; ^∗∗∗^*p* < 0.001. ns: not significant.

**Table 1:** General demographic characteristics of the patients at discharge for both groups ($\bar{x}\pm s$, *n* (%)).

Group	Gender		Age (year)	Course of disease (year)	Body weight (kg)	Stage of iron overload degree			Serum ferritin (*μ*g/L)
	Males	Females				IIA	IIIA	IIIB	
Control group (*n* = 74)	36 (48.65)	38 (51.35)	8.42 ± 1.09	3.45 ± 0.83	21.53 ± 9.20	20 (27.03)	26 (35.14)	28 (37.84)	2552.15 ± 611.10
Intervention group (*n* = 74)	42 (56.76)	32 (43.24)	8.60 ± 1.37	3.21 ± 0.95	21.81 ± 8.30	23 (31.08)	29 (39.19)	22 (29.73)	2528.35 ± 637.16
*t*/*χ*^2^/*Z*	0.976		0.884	1.637	0.194	-0.941			0.232
*P*	0.323		0.378	0.104	0.846	0.347			0.817

**Table 2:** Score of QLSCA between the two groups (point, $\bar{x}\pm s$).

Time	Control group (*n* = 74)	Intervention group (*n* = 74	*t*	*P*
Before intervention	78.75 ± 7.23	79.26 ± 6.73	0.444	0.658
12 weeks after intervention	91.45 ± 12.25	98.49 ± 13.48	3.325	0.001
24 weeks after intervention	100.19 ± 11.37	105.87 ± 10.52	3.154	0.002

RETRACTED

**Table 3:** Score of ESCA between the two groups (point, $\bar{x}\pm s$).

Time	Control group (*n* = 74)	Intervention group (*n* = 74)	*t*	*P*
Before intervention	89.26 ± 15.22	88.85 ± 14.69	0.167	0.868
12 weeks after intervention	102.45 ± 12.56	116.39 ± 13.51	6.501	<0.001
24 weeks after intervention	118.35 ± 11.54	128.62 ± 10.28	5.716	<0.001

**Table 4:** Score of medication compliance scale between the two groups (point, $\bar{x}\pm \text{s}$).

Time	Control group (*n* = 74)	Intervention group (*n* = 74)	*t*	*P*
Before intervention	19.15 ± 2.24	18.87 ± 3.32	0.601	0.548
12 weeks after intervention	21.58 ± 3.36	23.19 ± 3.47	2.867	0.005
24 weeks after intervention	23.68 ± 2.55	25.27 ± 2.48	3.845	<0.001

**Table 5:** Score of FAD (total function) between the two groups (point, $\bar{x}\pm \text{s}$).

Time	Control group (*n* = 74)	Intervention group (*n* = 74)	*t*	*P*
Before intervention	2.95 ± 0.58	3.01 ± 0.62	0.608	0.544
12 weeks after intervention	2.48 ± 0.32	2.25 ± 0.29	4.581	<0.001
24 weeks after intervention	2.21 ± 0.18	2.06 ± 0.13	5.811	<0.001

## Data Availability

The simulation experiment data used to support the findings of this study are available from the corresponding author upon request.
